# Biological Potential of Products Obtained from Palm Trees of the Genus *Syagrus*

**DOI:** 10.1155/2021/5580126

**Published:** 2021-08-19

**Authors:** Davi de Lacerda Coriolano, Maria Helena Menezes Estevam Alves, Isabella Macário Ferro Cavalcanti

**Affiliations:** ^1^Federal University of Pernambuco (UFPE), Laboratory of Immunopathology Keizo Asami (LIKA), Recife, Pernambuco, Brazil; ^2^Federal University of Pernambuco (UFPE), Laboratory of Microbiology and Immunology, Academic Center of Vitória (CAV), Vitória de Santo Antão, Pernambuco, Brazil

## Abstract

Medicinal plants have been used for centuries by communities worldwide, as they have diverse biological properties and are effective against numerous diseases. The genus *Syagrus* stands out for its versatility and for so many activities presented by these palm trees, mainly due to its rich chemical and fatty acid compositions. The genus has antibacterial potential, has antibiofilm, antiparasitic, antioxidant, prebiotic, antiulcerogenic, anticholinesterase, and hypoglycemic activities, and can produce biodiesel, amid others. Among all species, *Syagrus coronata* and *Syagrus romanzoffiana* stand out, presenting the greatest number of activities and applications. The secondary metabolites obtained from these palm trees present high activity even in low concentrations and can be used against infections and chronic diseases. Furthermore, these plants have been used in some communities for years and have presented healing properties, especially in inflammatory processes. Therefore, the *Syagrus* genus proves to be promising, which shows a lot of therapeutic potential.

## 1. Introduction for Genus *Syagrus*

Currently, medicinal plants and bioactive compounds have a major research focus because there are several reports on their biological properties, therefore leading to high demand for these plants [1]. They have been used for centuries by different communities around the world, and they have different biological properties and are effective against numerous diseases [2]. Commonly used in Chinese herbal medicine for disease prevention, treatment, and cure for thousands of years [3], as well as in Ancient Mesopotamia and Egypt, as reported in the Bible [4], these plants and their compounds had a substantial role in the treatment of several acute and chronic diseases throughout centuries [5].

According to the World Health Organization (WHO), the use of traditional medicine practices grows around the world, including herbal medicine as the only form of therapy [6]. The use of these plants appears mainly in the forms of extracts and oils; however, studies are applied to isolate molecules, understand and formulate herbal medicines to combat infectious and chronic diseases [7]. Besides the traditional communities, the pharmaceutical industry is widely using natural compounds in their formulations, as well as using biotechnology to produce bioactive molecules isolated from plants on a large scale, especially due to the fact that plants are safer, have a lower cost, and better availability [8].

The pharmacological potential of these plants is due to secondary plant metabolism, a set of metabolic processes responsible for the interactions with the environment and the production of secondary metabolites with diverse biological and physio-chemical properties, like phenolic compounds, organic acids, terpenes, alkaloids, among others [9]. These secondary metabolites are produced under specific abiotic stress and pathogenic attacks, thus the production of these chemicals is a form of protection to the plant [10, 11]. In addition to those plants and their secondary metabolites pharmacological properties, some plants used in traditional medicine are also exploited in their areas, such as biotechnology, for the production of biodiesel, enzymes, bioremediation, and others, therefore expanding the dimension to humanity's usage of plants [12–14].

Many genera of plants from the Arecaceae family all around the world have been used in traditional medicine and have shown biological activity. The genus *Butia* from the Arecaceae family and the subfamily Arecoideae is prevalent in southern Brazil, eastern Paraguay, northeastern Argentina, and in the northwest and southeast of Uruguay, and presents many properties, such as antibacterial, anti-inflammatory, and antioxidant activities [15]. The genus *Euterpe* from the Arecaceae family and the subfamily Arecoideae, found abundantly in Brazil, also shows various biological activities, such as anti-inflammatory, antioxidant, antimicrobial, antinociceptive, anticancer, and antiatherogenic, among others [16, 17]. The genus *Elaeis* also from the Arecaceae family is native to Africa and areas of South and Central America and also presents numerous activities, among them antiparasitic and wound-healing properties [18].

With greater prevalence of the Arecaceae family in South America and mainly in the north and northeast of Brazil, the *Syagrus* genus stands out for its versatility. This genus of palm trees has 65 species, 2 subspecies, 14 natural hybrids, and several applications [19]. Belonging to the family Arecaceae and the subfamily Arecoideae, the species of the genus *Syagrus* has great socioeconomic importance in tropical savanna flora. These palm trees can grow in several areas, such as tropical, humid subtropical, semiarid, and cerrado areas, showing a variety of habitat with different climates [19–21], this reflects the fact that these plants are used by many communities as a nutritional source [22], in addition to being considered a therapeutic option due to its antibacterial [23], antiparasitic [24], antioxidant [25], hypoglycemic [26] activities, and other promising actions of this genus.

Thus, this work is important and innovative because it is the first review that highlights the biological potential and pharmacological properties of palm trees from the genus *Syagrus* and their promising approaches to the development of new therapeutic alternatives.

### 1.1. Methodology and Strategies

The elaboration of this review was based on the following stages: identification of the theme and development of the guiding question; establishment of inclusion and exclusion criteria, analysis, and selection of articles; interpretation of data and results; and the writing of this paper. The guiding question was “What are the biological properties of genus *Syagrus* palm trees?” The inclusion criteria adopted were studies related to the proposed theme published in either Portuguese or English between 2005 and 2021, indexed on online databases, such as U.S. National Library of Medicine (PubMed), ScienceDirect, Scopus, and Scientific Electronic Library Online (SciELO). Both reviews and original articles were included. In turn, repeated studies, studies that do not address the proposed theme, incomplete studies, duplicates, and monographs were excluded.

After the literary search, 80 articles were selected using the inclusion and exclusion criteria. The analysis of the selected studies made it possible to identify variables, observations, and data that gathered the knowledge about the potential of *Syagrus* palm trees. Both the analysis and the relationship of the data extracted from these articles were developed descriptively, making it possible to count, observe, describe, classify, and organize the knowledge generated about *Syagrus* palm trees' properties.

## 2. Biological Properties of Plants of the *Syagrus* Genus

### 2.1. Antibacterial Activity

Bacterial infections are a major public health problem worldwide, especially due to the high levels of resistance to antimicrobials, consequently resulting in failure treatments, hospital readmissions or prolonged hospitalizations, high rates of morbidity and mortality, and high costs to health systems. With the phenomenon of bacterial resistance associated with little discovery of drugs, the search for new therapeutic options of low cost and greater efficacy has found space and strength in the study of natural products against sensitive and resistant bacterial strains, especially against *Staphylococcus aureus* [27–29].

Silveira et al. [30] studied the antibacterial activity of the fruit and almond extracts of *Syagrus oleracea*, popularly known as guariroba, and tested against *Staphylococcus aureus* ATCC 25923, *Pseudomonas aeruginosa* ATCC 27853, and *Escherichia coli* ATCC 25922, inhibiting bacterial growth up to 74% (Table 1). Hughes [23] analyzed the antimicrobial potential of *Syagrus coronata*, popularly known as ouricuri or licuri, evaluating its potential against *Bacillus cereus* CCMB 282, *S. aureus* CCMB 285, *S. aureus* CCMB 262 (resistant to streptomycin and dihydrostreptomycin), and *S. aureus* CCMB 263 (resistant to novobiocin) (Table 1). The extracts showed antibacterial activity with minimum inhibitory concentrations ranging from 190 to 3120 *μ*g/mL. This activity was probably related to the complex that phenolic compounds in the extracts formed with extracellular proteins of the bacterial membrane.

Bessa et al. [27] evaluated the activity of essential oil and commercial oil of *S. coronata* against the strain of *S. aureus* UFPEDA 02 and clinical isolates of methicillin-resistant *S. aureus* (MRSA) and methicillin-sensitive *S. aureus* (MSSA) (Table 1). Bacteriostatic and bactericidal effects were observed when both oils were tested in all of the samples, although a higher concentration of the commercial oil was required.

In the study conducted by Santos et al. [31], anti-*S. aureus* activity was also evaluated from the essential oil of *S. coronata* seeds, and similar results were observed for both *S. aureus* UFPEDA 02 strain, and multidrug-resistant *S. aureus* clinical isolates (Table 1). In this same study, an in vivo experiment with *Galleria mellonema* was performed, and it was observed that the treatment with essential oil of *S. coronata* in infected larvae increased the survival rate of the larvae by 60%. In addition, a reduction of 4 log CFU/mL in bacterial load was observed after 3 days of treatment. Therefore, evidencing the antibacterial potential of natural products extracted from plants of this genus, highlighting the anti-*S. aureus* activity from the essential oil of *S. coronata*, which is rich in compounds with this property, such as lauric, oleic, and linoleic acids [27].

The mechanism of action of both *S. coronata* and *S. oleracea* is not fully elucidated, but lauric acid, one of the main compounds in those plants, acts on the destruction of the cell membrane and interferes with cellular processes, such as signal transduction and transcription [32, 33]. Capric acid, also one of the main compounds in those plants, can damage the bacterial membrane due to its hydrophobicity, thereby facilitating the entrance of hydrogen ions from the extracellular environment and the complete inactivation of the bacterial cells [33, 34].

Besides that, *S. coronata* oil was proved to be safe when evaluated by biochemical, hematological, and histological parameters and did not demonstrate mutagenic nor genotoxic effects even in high doses [35].

### 2.2. Antibiofilm Activity

Biofilms are complexes composed of a set of bacteria encapsulated in an array of extracellular polymeric substances linked to biotic or abiotic surfaces. This system offers greater security, stability, oxygen, and nutrients to the microorganisms of this complex, thus protecting them from stress and increasing their survival potential [36]. This virulence factor is the main agent responsible for chronic infections because this persistence conferred by the biofilm results in treatment failure, making it necessary to apply new therapeutic approaches [37].

In the study of Santos [31], with the essential oil of *S. coronata* rich in dodecanoic acid, it was evaluated the activity of this oil against the biofilm of *S. aureus* UFPEDA 02. As a result, a significant reduction in the matrix was observed of biofilm only at concentrations of 312 and 624 *μ*g/mL; however, the viability of biofilm cells was significantly reduced at all concentrations tested, showing a reduction greater than 50% in the concentration of 156 *μ*g/mL and a reduction of almost 100% at concentrations of 624 and 1248 *μ*g/mL. In addition, changes in the cellular structure of *S. aureus* were also observed, as well as a loss of roughness in the multiple layers of the three-dimensional structure of the bacterial biofilm.

Another similar research performed by Junior [38] evaluated the antibiofilm activity of the essential oil of *S. coronata*, rich in dodecanoic, decanoic, and octanoic acids, against the *Proteus mirabilis* UFPEDA 737 isolate. Above 500 *μ*g/mL, the essential oil inhibited biofilm formation by more than 55%. The mechanism of action of *S. coronata* is not fully elucidated, but its main compounds lauric acid, capric acid, and caprylic acid affect cell membranes and bacterial adhesins, virulence genes, capsule production, and cell adhesion, respectively [39].

### 2.3. Antiparasitic Activity

Even in modern society, parasitic infections are still one of the world's public health problems, causing millions of deaths each year. Parasitic infections are considered as neglected tropical diseases, mainly because they mostly affect people in underdeveloped countries, where a large part of the population lives in a situation of social vulnerability. Many of these diseases have high cytotoxicity treatment so new therapeutic alternatives are needed to fight these infections [40, 41].

Leishmaniasis is an endemic parasitic infection caused by more than 20 species of Leishmania. Present in 97 countries, leishmaniasis affects more than 1.3 million people every year. This infection has three main forms: cutaneous leishmaniasis, visceral leishmaniasis, and mucocutaneous leishmaniasis [42]. The treatment of leishmaniasis is very problematic, due to the increase in parasitic resistance to currently used therapies, serious side effects, unsatisfactory results, and high cost of treatment [43].

Rodrigues et al. [24] analyzed the anti-*Leishmania amazonensis* activity of the aqueous polymeric extract of *S. coronata* rich in procyanidin. They tested the potential of this extract against the promastigote and amastigote forms of *L. amazonensis*. The extract of *S. coronata*, at a concentration of 50 *μ*g/mL, was able to inhibit the growth of promastigotes after 30 minutes and make 100% of the promastigotes unviable after 60 minutes. In addition, increased cell volume and membrane rupture were observed in the promastigotes treated with aqueous extract, suggesting that the extract of *S. coronata* induced osmotic dysregulation in *L. amazonensis* promastigotes (Figure 1). In the same study, the extract of *S. coronata* was also able to reduce the index of association between macrophages and amastigotes of *L. amazonensis*, with a concomitant increase in the production of nitric oxide (NO). When mouse peritoneal macrophages were pretreated with the extract at a concentration of 33 *μ*g/mL, the association index was reduced by 70.4%, and NO production increased by 158.3% when compared to the control. When the treatment was applied 24 hours after macrophage infection, the 33 *μ*g/mL of the crude aqueous extract was able to reduce the association index by 71% and increase NO production by 90.4%. Therefore, demonstrating the potential of using this plant as a leishmanicidal drug, mainly due to the increase in NO production, which potentiates the mechanisms of death of *L. amazonensis*.

Chagas disease or American trypanosomiasis is an anthropozoonosis caused by *Trypanosoma cruzi*. This infection is also considered a neglected tropical disease and is an important social and public health problem in Latin America. The number of people infected with *T. cruzi* in the world is substantial, being between 6 and 7 million people infected. The treatment of Chagas disease is effective in patients in the acute phase of the disease; however, when the person has been infected for a long period, the effectiveness of the medication decreases, and the treatment becomes ineffective. In addition, the drug can cause side and adverse effects due to its high cytotoxicity to mammalian cells [44, 45].

Souza et al. [46] evaluated the trypanocidal activity of the essential oil of *S. coronata* seeds. Their results showed that half of the maximal inhibitory concentration (IC_50_) for *T. cruzi* epimastigotes was 100.6 ± 38 *μ*g/mL, the IC_50_ for amastigotes was 408.33 ± 23.36 *μ*g/mL and the lethal concentration (LC_50_) for trypomastigotes was 182.49 ± 58.05 *μ*g/mL. Thus, it was demonstrated that the essential oil of *S. coronata* was able to inhibit the growth of epimastigotes and decrease the viability of trypomastigotes with moderately toxic concentrations.

### 2.4. Antioxidant Activity

In metabolisms, there are several oxidative processes necessary for cell survival. These processes result in the production of free radicals, which are involved in a series of regulatory processes, such as cell proliferation, apoptosis, and gene expression. However, in excess, these free radicals cause changes in protein structure, amino acid oxidation, DNA damaging, aging, and other harms. Therefore, in recent years there has been an increase in the demand for molecules and products that protect the individual against oxidative stress, and plants have been shown to be strong candidates due to their chemical compositions [47, 48].

Andrade et al. [49] studied the antioxidant activity of *Syagrus romanzoffiana*, popularly known as Jerivá. This property of the plant was evaluated using the *β*-carotene/linoleic acid method, which assesses the activity of inhibiting free radicals formed in lipid peroxidation, and ABTS and DPPH methods, which are related to the search for free radicals. Using 0.4 mL of extracts from the pulp and kernel cake of *S. romanzoffiana*, inhibition rates of oxidation were 97.00 ± 0.43% and 95.13 ± 0.7%, respectively, when the *β*-carotene method was applied. The ABTS method also demonstrated high antioxidant activity in the samples, all of which were greater than 100 *μ*M Trolox·g^−1^. Using 30 *μ*L of the pulp extract, a result of 2498.49 ± 186.7 *μ*M Trolox·g^−1^ was obtained. In the same concentration of the kernel cake extract, the result was lower, obtaining 1314.87 ± 29.78 *μ*M Trolox·g^−1^. In the DPPH method, the concentration necessary to reduce the amount of DPPH (EC₅₀) was measured. The best result once again was from the pulp extract of *S. romanzoffiana*, presenting an EC₅₀ = 96.97 ± 3.74 g fruit·g^−1^ DPPH, whereas the kernel cake extract showed EC₅₀ of 331.80 ± 3.95 g fruit·g^−1^ DPPH. The authors state that the large number of phenolic compounds in this oil may have contributed to this antioxidant activity [49].

According to Coimbra and Jorge [50], the antioxidant activity of Jerivá pulp oil can be justified by a large amount of *β*-carotene and tocopherols, with a total of 1219.01 ± 16.21 *μ*g/g for carotenoids and a total of 323.50 ± 7.85 mg/kg for tocopherols, with *α*-tocopherol being the most abundant (273.53 ± 4.79 mg/kg). Both compounds have proven antioxidant activity in vivo and in vitro. *β*-Carotene can function as a lipid scavenger and an oxygen extinguisher because of its unique structure of conjugated double bonds and ionone rings [51], and tocopherols can deactivate reactive oxygen species, inhibit protein oxidation, and prevent the propagation of lipid peroxidation by scavenging lipid peroxyl radicals [52], thus showing their potent antioxidant activity.

Belviso et al. [25] evaluated the antioxidant activity of *S. coronata* using the methods of DPPH and ABTS. The extract of toasted *S. coronata* seeds showed better antioxidant activity, presenting DPPH = 7.01 ± 0.23 *μ*M TE/g and ABTS = 5.31 ± 0.74 *μ*M TE/g, whereas the extract of raw seeds showed DPPH = 5.88 ± 0.16 *μ*M TE/ge ABTS = 4.07 ± 0.17 *μ*M TE/g.

The antioxidant activity of *S. oleracea* was also tested in the studies by Silva et al. [53] and Siqueira et al. [54]; however, the results were not as promising as those found in the two plants shown above. In the study by Silva [53], the EC₅₀ of *S. oleracea* extract in the DPPH test was 425.5 ± 1.9 *μ*g/mL, this result demonstrates low antioxidant activity. Siqueira et al.'s [54] obtained rate inhibition of oxidation by the ß-carotene method was 0.7 ± 0.1%/g, a very low rate.

### 2.5. Prebiotic Activity

Approximately 100 trillion microorganisms are inhabiting the human gastrointestinal tract. This microbiota present in the gastrointestinal system is part of a complex ecosystem that plays an important role in maintaining people's well-being and health [55]. Prebiotics are compounds selectively used by host microorganisms that can promote health benefits to the individual. They can be used as an energy source and stimulate the growth of microorganisms in the intestinal microbiota. Despite the benefits, the prebiotics available are not easily accessible, due to the high cost, so new alternatives are sought, such as the use of medicinal plants [49, 56].

Andrade et al. [49] studied the prebiotic potential of *S. romanzoffiana* pulp and kernel cake through the analysis of factors such as microbial growth, fermentation, and organic acids produced by the strains *Bifidobacterium lactis* BLC1, *Lactobacillus casei* BGP93, and *Lactobacillus acidophilus* LA3, in addition to of the pH change. The *S. romanzoffiana* pulp showed the best results, showing significant growth of 9.09 ± 0.09 log CFU/mL, 9.20 ± 0.11 log CFU/mL, and 8.76 ± 0.12 log CFU/mL for B. lactis, *L. casei*, and *L. acidophilus*, respectively. The greater growth of the probiotic strains was the result of the use of the carbon present in the *S. romanzoffiana* pulp as an energy source for bacteria. A greater decrease in pH was also observed after the administration of the *S. romanzoffiana* pulp, proving once again the probiotic potential of the plant, since a reduction in pH can be caused by the production of organic acids such as lactic, acetic acid, propionic, and butyric by bacteria during fermentation, thus indicating bacterial growth of probiotic strains and possible inhibition of the proliferation of pathogenic bacteria.

### 2.6. Antiulcerogenic Activity

Peptic ulcers are an increasingly common problem in the world population, affecting millions of people every year. They are lesions in the gastroduodenal mucosa, which cause frequent pain and gastrointestinal hemorrhage, resulting in loss of the patient's quality of life [57].

Silva and Parente [58] studied the antiulcerogenic activity of a galactomannoglucan extracted from the pulp of *S. oleracea*. In this in vivo experiment, male Swiss mice exposed to absolute ethanol, a substance that attacks the mucous membrane of the stomach, presented widespread and intense gastric hyperemia, in addition to thick lesions (control group). On the other hand, the group treated with galactomannoglucan extracted from *S. oleracea* before the exposition to absolute ethanol, had a stomach close to normal, with a great reduction in gastric hyperemia and formation of lesions after the administration of ethanol, thus evidencing the antiulcerogenic and gastroprotective activity of this natural compound (Figure 2). This gastroprotective activity was attributed to the chemical structure of galactomannoglucan, which is characterized by an initial chain of ß-D-galactose linked to (1–3) and terminal residues composed of *α*-D-glucose linked to (1–4) and is similar to antiulcerogenic polysaccharides that can induce mucus production.

### 2.7. Anticholinesterase Activity

Alzheimer's is a neurodegenerative disease that progressively deteriorates mental functions. In this disease, the cholinergic function is affected, like acetylcholine, a neurotransmitter responsible for conducting electrical impulses from one nerve cell to another, is reduced in quantity due to the rapid hydrolysis carried out by acetylcholinesterase. Therefore, cholinesterase inhibitors can be used in the treatment of this disease because they would inhibit the premature hydrolysis caused by acetylcholinesterase [59, 60].

El-Hawary et al. [61] evaluated the anticholinesterase activity of hydroalcoholic extracts of leaves and fruits of *S. romanzoffiana* in an in vivo experiment (Figure 3). The experiment was based on the administration of doses of 50 and 100 mg/kg.b.wt. of *S. romanzoffiana* extracts in rats for 2 months. Treatment with 50 mg/kg.b.wt. of the fruit extract resulted in a 21.5% reduction in acetylcholinesterase activity, whereas treatment with 100 mg/kg.b.wt. of this same extract resulted in a reduction of 26.5%. Treatment with 50 mg/kg.b.wt. of the extract of the leaves of the jerivá, resulted in a reduction of 22% in the activity of acetylcholinesterase, already the treatment with 100 mg/kg.b.wt. of this same extract resulted in a reduction of 29%. Both extracts showed significant reductions in cholinesterase activity, mainly due to the richness of fatty acids, flavonoids, and stilbenoids present in the extracts.

### 2.8. Hypoglycemic Activity

Diabetes mellitus is a metabolic disease characterized by an increase in blood glucose. It is a disorder that affects more than 400 million people worldwide and presents many health risks, which can cause microvascular and macrovascular complications, kidney failure, myocardial infarction, stroke, and the need to amputate limbs, thus reducing the quality and life expectancy of individuals. One of the alternatives for treating diabetes mellitus is to delay glucose absorption by inhibiting carbohydrate hydrolysis enzymes, such as *α*-glucosidase, and this inhibitory potential has been discovered in natural products [62, 63].

Lam et al. [26] evaluated the potential of *S. romanzoffiana* seed extract to inhibit *α*-glucosidase. As a result, it was observed that 10 *μ*g/mL of the ethanolic extract of *S. romanzoffiana* inhibited *α*-glucosidase by 55% and the butanoic fraction of this extract at the same concentration was able to inhibit even more (73%) (Figure 4). In addition, 8 compounds were identified in the extract and subsequently had their inhibitory activities evaluated, where 2 of them had excellent anti-*α*-glucosidase potential. The first isolated compound was the stilbene-phenylpropanoid 13-hydroxycompasinol A. This compound showed an inhibitory effect with an IC₅₀ of 6.5 *μ*M, and the second compound was the dimeric stilbenoid scirpusin C, which showed an even greater inhibitory effect, with an IC₅₀ of 4.9 *μ*M.

In the study of Lam and Lee [64], 6 other compounds extracted from *S. romanzoffiana* had their hypoglycemic activity evaluated, and 4 of them showed anti-*α*-glucosidase activity. *Syagrusins* A and B had ICs₅₀ of 16.9 and 23.7 *μ*M, respectively, 5-hydroxyapanol had IC₅₀ of 12.8 *μ*M, and the first phenylpropanoid had IC₅₀ of 10.7 *μ*M, thus, once again showing the potential that *S. romanzoffiana* extract and compounds have for the development of hypoglycemic drugs, especially stilbenoids.

### 2.9. Pharmacological Properties Suggested by Ethnobiological and Ethnopharmacological Studies

Ethnobiological and ethnopharmacological studies are greatly important for the discovery of new drugs of plant origin. These studies are based on research on the experiences of a community with the use of medicinal plants and their applications. From this, the most promising plants and genera are delimited, making the use of these plants more reliable and safer [65, 66].

Some researchers have already indicated the popular use of products of the *Syagrus* genus. In the study performed by Ribeiro et al. [67] in the northern microregion of Araguaia, in the state of Mato Grosso, the fruit of the *Syagrus comosa* (Mart.) plant, popularly known as bacuri, is used for conjunctivitis and *S. oleracea* for indigestion, diarrhea, and as an appetite stimulant. In the study performed by Rufino et al. [68] in a community near the Catimbau Valley National Park, municipality of Buíque, Pernambuco, was reported that *S. coronata* is used for the treatment of eye inflammation, mycoses, wound healing, and pain in the spine.

Junior, Ladio, and Albuquerque [69], in the community of Carão, municipality of Altinho, in the harsh region of Pernambuco, indicated that the plant *Syagrus cearensis*, popularly known as coco-catolé, had anti-inflammatory activity. Individuals in that community reported improvement after using *S. cearensis* for pain caused by cuts, swelling of wounds, redness, and itchy eyes. However, despite the use of these plants in these communities, experimental studies must be conducted to prove their effectiveness and better elucidate the mechanisms of action of these natural products.

### 2.10. Other Applications

In addition to the pharmacological properties already mentioned in this article, plants of the *Syagrus* genus still have other possible applications (Table 2) [13, 14, 70–80], mainly due to their chemical composition. The areas that stand out the most are biotechnology, for biodiesel production at an equal quality or better than the biodiesels on the market. Another success is in bioremediation, bringing fast, cheap, and efficient absorption of effluent materials.

## 3. Conclusion

*Syagrus* genus has a large group of palm trees rich in bioactive compounds, presenting several pharmacological properties that can be used from facing bacterial and parasitic infections to the treatment and/or prevention of chronic diseases such as diabetes and Alzheimer's disease. In addition, they show versatility to be used in other areas, such as the production of biodiesel, energy, enzymes, and among others. *Syagrus coronata* stands out when it comes to bacterial and parasitic infections, and *Syagrus romanzoffiana* stands out mostly against chronic diseases, showing anticholinesterase and anti *α*-glucosidase activity. In addition, they show versatility to be used in other areas, such as the production of biodiesel, energy, enzymes, and among others. However, despite demonstrating potential, further studies should be conducted to better elucidate the mechanism of action, pharmacokinetics, and possible side effects of these natural products.

## Figures and Tables

**Figure 1:** Mechanism of action of *S. coronata* extract against promastigote of Leishmania amazonensis (created with BioRender.com). Color indicates that *Syagrus coronata* aqueous extract increased cell volume and caused membrane rupture in the promastigotes due to osmotic dysregulation.

**Figure 2:** Gastroprotective action of galactomannoglucan extracted from *S. oleracea* (created with BioRender.com). Color indicates that Group 2 is treated with galactomannoglucan extracted from the pulp of *S. oleracea* and gets protected from ethanol action, but the control group treated only with water develops lesions and intense gastric hyperemia.

**Figure 3:** *S. romanzoffiana* extract slows acetylcholine hydrolysis (created with BioRender.com). Color indicates that *S. romanzoffiana* extract slows acetylcholine hydrolysis by inhibiting acetylcholinesterase action, consequently increasing the amount of acetylcholine and enabling the passage of acetylcholine.

**Figure 4:** Decreased glucose absorption by the *α*-glucosidase inhibition process caused by the extract of *S. romanzoffiana*, created with BioRender.com. Color indicates that the extract of *S. romanzoffiana* inhibits carbohydrate hydrolysis by the inhibition of *α*-glucosidase, thus decreasing glucose absorption.

**Table 1:** Antibacterial activity of compounds extracted from *Syagrus* genus.

Plant	Popular name	Natural compounds	Bacteria	References
*Syagrus oleracea*	Guariroba	Hexane fraction of the epicarp/mesocarp	*Staphylococcus aureus* ATCC 25923 *Pseudomonas aeruginosa* ATCC 27853 *Escherichia coli* ATCC 25922	[27]

*Syagrus coronate*	Ouricuri or licuri	Aqueous inflorescence extract	*Bacillus cereus* CCMB 282 *S. aureus* CCMB 262 *S. aureus* CCMB 263 *S. aureus* CCMB 285	[20]

*Syagrus coronate*	Ouricuri or licuri	Essential oil and commercial oil extracted from the seeds	*S. aureus* UFPEDA 02 Methicillin-resistant *S. aureus* (MRSA) clinical isolate Methicillin-sensitive *S. aureus* (MSSA) clinical isolate	[24]

*Syagrus coronata*	Ouricuri or licuri	Essential oil extracted from the seeds	*S. aureus* UFPEDA 02 Multidrug-resistant *S. aureus*	[28]

**Table 2:** Possible applications of plants of the *Syagrus* genus.

Application area	Possible application	Product	Plant	Popular name	References
Nanotechnology	Transport of amphotericin B for topical application	Microemulsion with oil	*Syagrus cearensis*	Coco-catolé	[65]
Insecticides	Promotion of the death of *Aedes aegypti* larvae, as well as reduction in oviposition	Volatile oil	*Syagrus coronata*	Ouricuri or licuri	[66]

Biotechnology	Biodiesel production	Crude walnut oil	*Syagrus coronata*	Ouricuri or licuri	[67]
	Biodiesel and bio oil production	Walnut	*Syagrus coronata*	Ouricuri or licuri	[12]
	Substrate for mycelium bioconversion basidiomas and for ligninolytic enzyme production by *Ganoderma lucidum*	Agricultural waste (fruit peels, leaves, and bracts)	*Syagrus coronata*	Ouricuri or licuri	[13]
	Energy production	Nutshell	*Syagrus coronata*	Ouricuri or licuri	[68]
	Biodiesel production	Oil from seeds	*Syagrus romanzoffiana*	Jerivá	[69]
	Biodiesel production	Almonds	*Syagrus cearensis*	Coco-catolé	[70]

Bioremediation	Bioremoval of methylene blue from aqueous solutions	Fibers	*Syagrus coronata*	Ouricuri or licuri	[71]
	Bioremoval of methylene blue from aqueous solutions	Activated carbon obtained from the endocarp	*Syagrus oleracea*	Guariroba	[72]
	Bioremoval of Cu (II) from aqueous solutions	Coal obtained from the fruit peel	*Syagrus coronata*	Ouricuri or licuri	[73]
	Biosorption of ciprofloxacin from aquatic effluents	Activated carbon obtained from the endocarp	*Syagrus romanzoffiana*	Jerivá	[74]
	Biosorption of diclofenac in aquatic effluents	Material using charcoal from the endocarp	*Syagrus coronata*	Ouricuri or licuri	[75]

## Data Availability

This review article was carried out by searching for review and original articles related to the proposed theme available on online databases, such as U.S. National Library of Medicine (PubMed), ScienceDirect, Scopus, and Scientific Electronic Library Online (SciELO), published in either Portuguese or English between 2005 and 2021.
